# Awareness of Birth Preparedness and Complication Readiness in Southeastern Nigeria

**DOI:** 10.5402/2011/560641

**Published:** 2011-07-25

**Authors:** John E. Ekabua, Kufre J. Ekabua, Patience Odusolu, Thomas U. Agan, Christopher U. Iklaki, Aniekan J. Etokidem

**Affiliations:** ^1^Department of Obstetrics & Gynecology, University of Calabar Teaching Hospital, Calabar P.M.B 1278, Calabar, Cross River State, Nigeria; ^2^Department of Community Medicine, University of Calabar Teaching Hospital, Calabar P.M.B 1278, Calabar, Cross River State, Nigeria

## Abstract

The aims of this study are to assess the awareness and intention to use maternity services. This was a multicentric study involving 800 women. Educational status was the best predictor of awareness of birth preparedness (*P* = 0.0029), but not a good predictor of intention to attend four antenatal clinic sessions (*P* = 0.449). Parity was a better predictor of knowledge of severe vaginal bleeding as a key danger sign during pregnancy than educational level (*P* = 0.0009 and *P* = 0.3849, resp.). Plan to identify a means of transport to the place of childbirth was related to greater awareness of birth preparedness (*χ* ^2^ = 0.3255; *P* = 0.5683). Parity was a highly significant predictor (*P* = 0.0089) of planning to save money. Planning to save money for childbirth was associated with greater awareness of community financial support system (*χ* ^2^ = 0.8602; *P* = 0.3536). Access to skilled birth attendance should be promoted.

## 1. Introduction

The principle and practice of birth preparedness and complication readiness (BP/CR) in a third world setting where there is prevailing illiteracy, inefficient infrastructure, poor transport system, and unpredictable access to skilled care provider have the potential of reducing the existing high maternal and neonatal morbidity and mortality rates. BP/CR promotes skilled care for all births and encourages decision making before the onset of labor [1]. The BP/CR matrix raises awareness of danger signs, thereby improving problem recognition and reducing delay in deciding to seek care [2]. It provides information on appropriate sources of care (promoters and facilities) making the care-seeking process more efficient. It also encourages households and communities to set aside money for transport and service fees, avoiding delays in reaching care caused by the search for funds. However, antenatal care in Nigeria is provided along the lines of the traditional approach based on risk assessment and not on the goal-oriented interventions of focused antenatal care, which include BP/CR [3]. The study is a needs assessment designed to determine the level of awareness, attitude and behavior of women to birth preparedness, and complication readiness.

## 2. Method

### 2.1. Study Area

This cross-sectional, multicentric descriptive study was carried out in Calabar and Biase Local Government Areas of Cross River State, Nigeria. Calabar is the capital of Cross River State. It is made up of two Local Government Areas (LGAs) and 22 geopolitical wards. The total population for this area is 418,652 with majority of the workforce being in government employment or involved in small-scale business ventures. The area hosts a Teaching Hospital, one General Hospital, several maternal and child health centers, and several private hospitals. Biase Local Government Area has an area of 1,310 km² and a population of 169,183. Apart from Akpet Central, which is the local government headquarters, the rest of the area is rural.

### 2.2. Subjects and Method

A cross-sectional survey of 800 women, who gave birth between 1st January and 31st December 2008, attending two urban (Calabar) and two rural (Biase Local Government Area) maternal and child health clinics in Cross River State, Nigeria, was undertaken between January and April, 2009. Informed oral consent was sought and obtained from participants before inclusion in the study. After due explanation of the study and necessary clarifications of issues raised, the field assistants distributed the questionnaires to the women surveyed. The women were assured of confidentiality and that their names will not be published in the report. The self-administered structured questionnaires were retrieved after two weeks at each study center by field assistants. The study design fulfilled the requirements set by the ethics committee of the Cross River State Ministry of Health. The number of questionnaires returned was 776, giving a survey response rate of 97%. Incorrect or incomplete entries on the questionnaires were excluded from analysis. Data obtained were analyzed using epi info 2002 software, with logistic regression/test of association performed. Information obtained included sociodemographic characteristics; history of last confinement; danger signs in last pregnancy; awareness of birth preparedness and key danger signs; intention of service use; and knowledge of available community support systems. Knowledge of key danger signs and available community support system were assessed according to the proportion of women who correctly answered the relevant questions as follows: *excellent*: > 80%; *good*: 60% to < 80%; *poor*: > 30% but <60%; *very poor:* < 30%. 

For clarity, some terms used in this paper are defined as follows.

- *Birth preparedness and complication readiness (BP/CR) [2]* is the process of planning for normal birth and anticipating the actions needed in case of an emergency.
- *BP/CR matrix [2]* delineates the roles (plans/actions) of policymakers, facility managers, care providers, communities, families, and women in ensuring that women and newborns receive timely appropriate and effective care.
- *Skilled care provider/attendant [4]* is a professional caregiver who has the knowledge and skills to manage labor, childbirth, and postpartum period; recognize complications; diagnose, manage, or refer woman or newborn to a higher level of care if complications occur that require interventions beyond current caregiver's competence.
- *Postpartum period* is defined as beginning after delivery of the placenta to 6 weeks after birth.
- *Newborn/neonatal period* refers to the first 7 days of the newborn's life.
- *Risk factor [5]* is defined as one link in a chain of associations leading to an illness or an indicator of link; and is identifiable prior to the event it predicts.
- *Community emergency response mechanism [6]* the community is defined as having an emergency response mechanism if all of the following systems are in place: identification of pregnant women, finance, transportation, blood donation, and at least one contact person responsible for linking these systems to the women in need.

## 3. Results

**Table 1**

The sociodemographic profile of women surveyed showed that 79.4% were aged 20–39 years; 78.9% were married; 54.8% had secondary education; 61.9% were para 2–4.

**Tables 2 and 3**

The proportion of women residing in the rural area was 55.1%. Hospital delivery was recorded in 48.8%. The commonest means of transport in last confinement was the motorcycle (64.7%). The commonest danger signs experienced were as follows: in last pregnancy, prolonged labor (22.4%); in the baby, stillbirth (5.2%); after delivery, severe vaginal bleeding (19.1%). Log regression data showed that residence was a good predictor of the place of last confinement. Women who resided in urban areas were more likely to deliver in the hospital than those who resided in rural areas (*χ* ^2^ = 24.038; *P* < 0.0001). None of the women delivering outside the hospital received skilled attention. Women who were in labor for more than 24 hours were more likely to undergo caesarean section than those who were in labor for less than 12 hours; however, this difference was not statistically significant (*χ* ^2^ = 4.5440; *P* = 0.3374). Women who were in labor for more than 24 hours were more likely to notice difficult/fast breathing in their babies than those who were in labor for 12 to 24 hours; however, this difference was not statistically significant (*χ* ^2^ = 1.4217; *P* = 0.4912).

**Table 4**

Although awareness of the concept of birth preparedness was high (70.6%), knowledge of specific key danger signs was poor. Logistic regression analysis showed that of the four variables, age, educational status, marital status, and parity, educational status was the best predictor of awareness of the concept of birth preparedness (*P* = 0.5477; 0.0029; 0.6455; 0.4433, resp.). The place of residence, urban or rural, was not a good predictor of awareness of birth preparedness (*χ* ^2^ = 0.3316; *P* = 0.5646). Parity was a better predictor of knowledge of severe vaginal bleeding as a key danger sign during pregnancy than educational level (*P* = 0.0009 and *P* = 0.3849, resp.).

**Table 5**

Intention and behavior as regards plan to use maternity services during pregnancy and access skilled attendance in childbirth was generally positive (ranging from 69.5% to 83.5%). However, log regression analysis showed that educational level, marital status and parity were not good predictors of intention and behavior, especially regarding plan to attend at least four antenatal clinic (ANC) visits with a skilled provider (*P* = 0.449; 0.1286 and 0.9765, resp.). Those who were aware of birth preparedness were more likely to plan to identify mode of transport to the place of childbirth than those who were not aware. This difference was not statistically significant (  *χ* ^2^ = 0.3255; *P* = 0.5683). When planning to save money for childbirth was regressed on marital status, educational level, awareness of birth preparedness, and parity, it was observed that parity was a highly significant predictor (*P* = 0.0089) of planning to save money followed by awareness of birth preparedness (*P* = 0.0101). Marital status and level of education were not good predictors of planning to save money for childbirth (*P* = 0.2394, 0.2013, resp.). Women who planned to save money for child birth were more aware of community financial support system than those who did not plan to save money. This difference was not statistically significant (*χ* ^2^ = 0.8602; *P* = 0.3536). Knowledge of availability of community support systems was very poor among women surveyed.

## 4. Discussion

Birth preparedness and complication readiness (BP/CR) is the process of planning for normal birth and anticipating the actions needed in case of an emergency [2]. Responsibility for BP/CR must be shared among all safe motherhood stakeholders—policymakers, facility managers, providers, communities, families, and women—because a coordinated effort is needed to reduce the delays that contribute to maternal and newborn deaths. Women and newborns need timely access to skilled care during pregnancy, childbirth, and the postpartum/newborn period. Too often, however, their access to care is impeded by delays—delays in deciding to seek care, delays in reaching care, and delays in receiving care [7]. These delays have many causes, including logistical and financial concerns, unsupportive policies, and gaps in services, as well as inadequate community and family awareness and knowledge about maternal and newborn health issues [2]. This study focuses on the individual woman's awareness of BP/CR and her intention/behavior toward eliminating delay when deciding to seek care.

The rural population of Nigeria in 2008 was put at 52% of the total [8]. There was a slight preponderance of respondents in this study residing in rural areas. About 50% of women in this study had hospital delivery. Women who resided in urban areas were more likely to deliver in the hospital than those who resided in rural areas (*P* < 0.0001). This is to be expected because in Nigeria, the inverse care law operates. Provision of social amenities, including medical care, is concentrated in urban centers. According to the Nigeria demographic and health survey, 66% of Nigerian women deliver at home [9]. This is a dangerous trend that needs urgent attention, if the prevailing high maternal mortality and morbidity in the country is to be reversed. None of the women who delivered outside the hospital, in this study, received skilled attention. As seen in this study, women experienced emergency situations in the last pregnancy from reported danger signs that needed skilled intervention, such as prolonged labor, stillbirths, and severe vaginal bleeding after delivery. Maternal mortality resulting from the reported danger signs is beyond the scope of this study. Women who were in labor for more than 24 hours were more likely to undergo caesarean section than those who were in labor for less than 12 hours. Also, women who were in labor for more than 24 hours were more likely to notice difficult/fast breathing in their babies than those who were in labor for 12 to 24 hours. These were situations needing skilled attendance, so as to reduce morbidity and mortality in mother and baby. 

Distance was an issue in seeking skilled attention, with up to half of the women having to travel up to 2 km or more to reach the nearest hospital. In a Nigerian study, 41% of the mothers who did not deliver in hospital explained that they could not afford the hospital bill, and 31% said they had transportation challenges [10]. The commonest means of transport in the last confinement was the motorcycle. We have shown in a previous study that this is a dangerous means of transportation for pregnant women, because the risk of serious morbidity following an accident is high [11]. A study from Nepal showed that a distance of more than one hour to the maternity hospital was statistically associated with an increased risk of home delivery [12].

The awareness of the concept of birth preparedness in this study was unexpectedly high. This is because the goal-oriented interventions of focused antenatal care [13], which include BP/CR, are yet to be implemented in the Cross River State maternity services. Pregnant women are cared for on the basis of risk assessment in the traditional approach to antenatal care [3]. They are not usually counseled on the importance of recognizing danger signs, saving money for childbirth, and identifying a means of transport before delivery, among other issues of BP/CR matrix. That is why there is a disparity between awareness of the concept of birth preparedness and knowledge of specific danger signs in pregnancy, labor, and after childbirth. The knowledge of danger signs was rated to be poor in this study. Logistic regression analysis showed that educational status was the best predictor of awareness of the concept of birth preparedness. However, there was no association between awareness of birth preparedness and place of residence. Contrary to expectation, place of residence (urban or rural) was not a good predictor of awareness of birth preparedness. This is because educational status was the best predictor of awareness of birth preparedness, and the more educated women usually reside in the urban areas. Parity was a better predictor of knowledge of severe vaginal bleeding as a key danger sign during pregnancy than educational level. This can be explained by the fact that severe vaginal bleeding was a reported danger sign by women in the last pregnancy, and this experience was related more to parity than educational status. 

In order for awareness of BP/CR to result in improved access to skilled attendance, there has to be action plan and service use. The type of action plan undertaken by women in preparation for childbirth will depend on right intention and appropriate behavior. Although this study showed that intention and plan to use maternity services were positive; educational level, marital status and parity were not good predictors of intention and behavior, especially regarding plan to attend at least four ANC visits with a skilled provider. This is an unfortunate finding as studies have shown that women who attend ANC are more likely to deliver in hospital [12]. Also, about 20% of women in this study experienced emergency situations in the last confinement that needed skilled intervention. However, none of the demographic variables analyzed was associated with a significant intention to seek skilled attendance in future pregnancies. Awareness of birth preparedness was associated with a plan to identify a mode of transport to the place of childbirth before onset of labor. Transportation is a challenge in Nigeria, especially to pregnant women [10, 11]. Road networks are poor in many urban areas and virtually nonexistent in rural areas. In addition, the transport system is inefficient and not always available when needed. That is why the establishment of a community support system with regard to transportation is a desirable measure to assist pregnant women, especially when an emergency arises. Unfortunately, knowledge of such support system in the community was very poor. Financial constraint in Nigeria is a major obstacle to accessing skilled attendance in pregnancy [10, 14]. It is therefore appropriate for pregnant women to save money for childbirth and to be able to access emergency funds when needed. Parity was a highly significant predictor of planning to save money followed by awareness of birth preparedness. This finding may be related to past experience of danger signs in pregnancy and childbirth. Also, intention to save money was associated with knowledge of community financial support system. This is a step in the right direction and should be encouraged. The existence of community-level systems to provide emergency funds, transport, and blood donors, is vital in promoting maternal and newborn survival [6]. Community leadership therefore has an important role to play in removing barriers in deciding to seek care and improving access to a skilled care provider/attendant for women and their newborn babies. An emergency response system must be put in place and made known to the public. If women living in a community are ignorant of the existence of these emergency response systems, then they are unlikely to use and benefit from them. Also a system of identifying pregnant women through community-based health promoters will ensure that support/help is given when needed.

## 5. Conclusion

Although awareness of the concept of birth preparedness was high, recognition of key danger signs in pregnancy was poor. Proportion of births attended to by skilled attendant was low. Educational level, marital status, and parity were not good predictors of intention to attend at least four ANC visits with a skilled provider. The knowledge of available community support systems was very poor. 

Based on these findings, it is recommended that

- birth preparedness and complication readiness should be made an integral part of maternal and child health services in the state, to enable women to recognize danger signs and access a skilled caregiver in pregnancy;
- an emergency response system at the community level to provide emergency funds, transport, and blood donors must be put in place and made known to the public.

It is believed that with the removal of delays in decision to seek care and timely access to skilled attendance, the prevailing high maternal/infant morbidity and mortality in Nigeria can be reduced to acceptable limits.

## Figures and Tables

**Table 1:** Sociodemographic characteristics.

Variable (*n* = number)	Number	Percent (%)
Age group (*n* = 760)		
<20 years	72	9.5
20–39	604	79.4
40–49	84	11.1

Marital status (*n* = 740)		
Never married	120	16.2
Married	584	78.9
Widow	12	1.6
Separated/divorced	24	3.2

Educational status (*n* = 744)		
No formal education	28	3.8
Primary education	204	27.4
Secondary education	408	54.8
Tertiary education	104	14.0

Parity (*n* = 724)		
1	160	22.1
2–4	448	61.9
>4	116	16.0

**Table 2:** History of last confinement.

History/event	Frequency	Percent (%)
Residence (*n* = 748)		
Urban	336	44.9
Rural	412	55.1

Place of last confinement (760)		
Hospital	368	48.4
Church	128	16.8
TBA	148	19.5
Home	116	15.3

Approximate distance from hospital (*n* = 696)		
<2 km	344	49.5
2–5 km	296	42.5
>5 km	56	8.0

Means of transport (*n* = 736)		
Taxi	72	9.8
Bus	44	6.0
Motor cycle	476	64.7
Boat	8	1.1
Trekking	124	16.8
Others	12	1.6
Non response	72	9.8

Duration of labour (*n* = 736)		
<12 hours	468	63.6
12–24 hours	204	27.7
>24 hours	64	8.7

Mode of delivery (*n* = 716)		
Vaginal	620	86.6
Episiotomy	32	4.5
Caesarean section	64	8.9
Instrumental	0	0.0

**Table 3:** Danger signs experienced in last pregnancy.

Variable	Frequency	Percent (%)
Danger signs during pregnancy		
Severe vaginal bleeding (*n* = 760)	84	11.1
Swollen hands and feet (*n* = 760)	96	12.6
Blurred vision (*n* = 752)	104	13.8
Prolonged labor (*n* = 768)	172	22.4
Convulsions (*n* = 752)	32	4.3
Retained placenta (*n* = 760)	56	7.4

Problems with baby		
Stillborn (*n* = 764)	40	5.2
Died within 7 days (*n* = 760)	20	2.6
Convulsions/spasms/rigidity (*n* = 760)	16	2.1
Difficult/fast breathing (*n* = 764)	32	4.2
Very small baby (*n* = 756)	28	3.7
Lethargy/unconsciousness (*n* = 756)	16	2.1

Danger signs after delivery		
Severe vaginal bleeding (*n* = 752)	144	19.1
Foul lochia (*n* = 744)	12	1.6
High fever (*n* = 720)	40	5.6

**Table 4:** Knowledge of specific danger signs.

Knowledge of variable	Frequency	Percent (%)
Awareness of birth preparedness (*n* = 680)	480	70.6

Key danger signs during pregnancy		
Severe vaginal bleeding (*n* = 744)	360	48.8
Swollen hands and face (*n* = 732)	376	51.4
Blurred vision (*n* = 740)	320	43.2

Key danger signs during labor and childbirth		
Severe vaginal bleeding (*n* = 756)	444	58.7
Prolonged labor (>12 hours) (*n* = 756)	396	52.4
Convulsion (*n* = 748)	260	34.8
Retained placenta (*n* = 740)	352	47.6

Key danger signs during postpartum period		
Severe vaginal bleeding (*n* = 760)	408	53.7
Foul lochia (*n* = 744)	244	32.8
High fever (*n* = 752)	356	47.3

Key danger signs in newborn		
Convulsions/spasms/rigidity (*n* = 748)	312	41.7
Difficulty/fast breathing (*n* = 748)	372	49.7
Very small baby (*n* = 740)	308	41.6
Lethargy/unconsciousness (*n* = 736)	160	21.7

**Table 5:** Complication readiness: service use and planning actions.

Intention and behavior	Frequency	Percentage (%)
Plan to attend at least 4 ANC visits with skilled provider (*n* = 696)	484	69.5

Plan to attend first ANC with skilled provider in first trimester (*n* = 680)	484	71.2

Plan to give birth with skilled attendant (*n* = 732)	580	79.2

Plan to save money for childbirth (*n* = 704)	564	80.1

Plan to identify mode of transport to place of childbirth (*n* = 776)	648	83.5

Knowledge of availability of community support systems (*n* = 736)		
Financial support system	148	20.1
Transport system	176	23.9
Blood donor system	24	3.3
